This article has been retracted.

# Perinatal Exposure to Bisphenol-A Impairs Spatial Memory through Upregulation of Neurexin1 and Neuroligin3 Expression in Male Mouse Brain

**DOI:** 10.1371/journal.pone.0110482

**Published:** 2014-10-17

**Authors:** Dhiraj Kumar, Mahendra Kumar Thakur

**Affiliations:** Biochemistry and Molecular Biology Laboratory, Brain Research Centre, Department of Zoology, Banaras Hindu University, Varanasi, India; Radboud University, Netherlands

## Abstract

Bisphenol-A (BPA), a well known endocrine disruptor, impairs learning and memory in rodents. However, the underlying molecular mechanism of BPA induced impairment in learning and memory is not well known. As synaptic plasticity is the cellular basis of memory, the present study investigated the effect of perinatal exposure to BPA on the expression of synaptic proteins neurexin1 (Nrxn1) and neuroligin3 (Nlgn3), dendritic spine density and spatial memory in postnatal male mice. The pregnant mice were orally administered BPA (50 µg/kgbw/d) from gestation day (GD) 7 to postnatal day (PND) 21 and sesame oil was used as a vehicle control. In Morris water maze (MWM) test, BPA extended the escape latency time to locate the hidden platform in 8 weeks male mice. RT-PCR and Immunoblotting results showed significant upregulation of Nrxn1 and Nlgn3 expression in both cerebral cortex and hippocampus of 3 and 8 weeks male mice. This was further substantiated by *in-situ* hybridization and immunofluorescence techniques. BPA also significantly increased the density of dendritic spines in both regions, as analyzed by rapid Golgi staining. Thus our data suggest that perinatal exposure to BPA impairs spatial memory through upregulation of expression of synaptic proteins Nrxn1 and Nlgn3 and increased dendritic spine density in cerebral cortex and hippocampus of postnatal male mice.

## Introduction

Bisphenol-A, a synthetic endocrine disrupting compound, leaches from polycarbonate plastics and reusable water bottle [1], [2]. It acts as either estrogen receptor agonist or antagonist and mediates its effects through steroid receptors pathways [3], [4], [5], [6]. It alters steroid hormone synthesis and clearance, receptor expression and gene activity in the target tissue [7], [8]. Moreover, gonadal hormones play an important role in the sexual differentiation of brain and behavior pattern during a critical period of development [9]. As the developing brain is highly sensitive to gonadal hormones, it becomes vulnerable to endocrine disrupting chemical like BPA [10]. Hence exposure to BPA influences brain development leading to pathologies and behavioral problems [11], [12]. Particularly in rodents, it affects the exploratory behavior [13], sociosexual behavior [14], anxiety level [15], [16] and impairs learning and memory [17], [18].

Learning and memory is directly related to synaptic plasticity of neuronal circuit in brain, mainly in hippocampus. The synaptic plasticity is enhanced by estrogen through increase in synaptogenesis, neuronal network connectivity and synaptic transmission [19], [20]. In ovariectomized rats, BPA was found to inhibit the estradiol induced hippocampal synaptogenesis [21]. During neonatal development, BPA enhanced the dendritic growth in cerebral purkinje cell and dendritic spine density in hypothalamic neurons of rats [22], [23]. Moreover, BPA exposure to rat hippocampal neurons in culture increased the motility and density of dendritic filopodia [24].

In mature nervous system, synapses form elegantly precise connections necessary for neural processing and function. However, the developing nervous system is characterized by crude synaptic wiring that must undergo a significant degree of remodeling through synaptic pruning to eliminate exuberant synaptic connections while maintaining the others [25]. The pattern of synaptic connectivity established during development critically determines the function of brain. The assembly of individual synapse is particularly mediated by bidirectional signaling between the pre and postsynaptic neurons [26], [27]. Synaptic cell adhesion molecules including neurexins (Nrxns) and neuroligins (Nlgns) control recognition events between pre and post synaptic neurons for orchestrating the structural organization of synaptic junctions [28], [29]. Nlgns form trans-synaptic complexes with presynaptic Nrxns [30] and play an important role in differentiation, maturation and stabilization of both excitatory and inhibitory synapses [31], [32], [33], [34]. Nlgn1 is found in excitatory synapses [35] and Nlgn2 in inhibitory synapses [34], whereas Nlgn3 in both [3]. Moreover, Nrxns/Nlgns interaction is involved in neuronal plasticity mechanism and predicted to influence the excitatory/inhibitory synapse ratio in brain [36], [37], [38].

However, it is not known whether exposure to BPA impairs learning and memory through alteration in the expression of synaptic proteins Nrxn1 and Nlgn3 and the density of dendritic spines. Therefore, we have investigated the effect of perinatal exposure to BPA in 3 and 8 weeks male mice. The effect was measured by behavioral test (MWM), expression of synaptic proteins Nrxn1 and Nlgn3 at mRNA and protein level, and evaluation of dendritic spine density by rapid Golgi staining technique.

## Experimental Procedure

This research was approved by the Central Animal Ethical Committee, Institute of Medical Sciences, Banaras Hindu University, Varanasi, India (Approval No.- CAEC/261).

### Animals

The inbred Swiss albino mice were maintained under a 12∶12 h light-dark cycle (light period 7∶00 am to 7∶00 pm) at 23–24°C in the animal house of Department of Zoology, Banaras Hindu University, Varanasi, India. They were provided food and water *ad libitum*. The mating (female: male, 2∶1) was set in the evening and the vaginal plug was examined next morning. The plug positive mice were designated gestational day (GD) 0 and pregnant mice were placed in a cage (one mouse in each cage). The mice were handled and used according to the guidelines of the institutional animal ethical committee, Banaras Hindu University, Varanasi, India.

### Treatment

The pregnant mice were orally administered BPA (99.8% pure, Sigma Aldrich, USA) dissolved in sesame oil (50 µg/kgbw/d) by gavages from GD 7 to PND 21 with care to avoid stress. This dose of BPA is in the range of low dose [39], [40] and has been used for mice by many investigators [41], [42], [43]. The control mice were administered sesame oil for the same duration. For each group of BPA and control, 10 pregnant mice were used. BPA and sesame oil were administered between 8∶30 am to 9∶30 am each day. The oral route of BPA administration was chosen to mimic the actual path of exposure to the wild life and human. After parturition, the pups were counted and culled to 8–10 pups/litter. On PND7, the sex of pups was individually identified based on anogenital distance [44] and equal number of both sexes was maintained with each mother. On PND 21, pups were weaned, housed in separate cages and allowed to grow to 8 weeks. Male mice of 8 weeks were used for spatial memory test in MWM task. The cerebral cortex and hippocampus were dissected out from 3 and 8 weeks male mice (n = 3×3 mice/group) for analyzing the expression of synaptic proteins Nrxn1 and Nlgn3. Furthermore, the whole brain from both age groups was processed for sectioning by cryostat for immunofluorescence and *in-situ* hybridization and by vibratome for rapid Golgi staining studies.

### Morris Water Maze Test

The MWM test, a well established and standard technique for evaluating the memory of rodents, was used as described earlier [45] with some modifications. The water maze consisted of a black circular pool (100 cm in diameter, 55 cm in height) filled with water to a depth of 26 cm (23–25°C). A submerged flexi glass platform was located at fixed (target) quadrant below 1 cm water level all through the experiment. The maze was divided into four equal quadrants: northwest (NW), northeast (NE), southwest (SW) and southeast (SE). Visual cues of cardboards of different shapes (round, square, triangle and star) and colors were placed on the cylindrical tank wall corresponding to quadrant corners. The established parameters like position and cues were maintained throughout the experiments. MWM test was conducted between 11∶00 am to 1∶00 pm to avoid the effect of diurnal variation. Test was conducted for 8 days and each day two consecutive tests were performed to check the effect of BPA in 8 weeks male mice. Maximum latency time was set as 60 s. If the mice failed to find the platform within 60 s, it was guided towards the platform and allowed to rest there for 15 s. On 9^th^ day, a probe test was conducted by removing the platform and noting the time spent in the target quadrant. A video camera was mounted above the centre of the maze and activity of mice was recorded for 60 s. The escape latency time during test and time spent in target quadrant during probe trial for each mouse was analyzed using ANY-maze software (Microsoft version 4.84, USA).

### Semiquantitative Reverse Transcriptase Polymerase Chain Reaction (RT-PCR)

Total RNA was isolated from the cerebral cortex and hippocampus of 3 and 8 weeks male mice using the TRI Reagent kit (Sigma-Aldrich, USA) according to the manufacturer’s instruction. It was estimated by taking absorbance at 260 nm and RNA sample with A_260/280_ of 1.8 was used. RNA from both ages was resolved on 1.2% agarose formaldehyde gel to check its integrity by ethidium bromide staining of 18S and 28S rRNA. For cDNA synthesis, 3 µg of total RNA and 200 ng random hexamer (Fermentas International Inc, Canada) were mixed in 11 µl reaction volume and denatured at 70°C for 5 min. Further, 2 µl of 10x reaction buffer, 2 µl of 10 mM dNTP mix and 20 U of RNase inhibitor (New England Biolabs, USA) were added, the volume was made up to 19 µl and incubated at 25°C for 5 min. Thereafter, 200 U of M-MuLv reverse transcriptase (New England Biolabs, USA) was added, and the tube was incubated first at 25°C for 10 min and then at 42°C for 1 h in a thermal cycler (Applied Biosystem, USA). The reaction was terminated by heating at 70°C for 10 min and the resulting cDNA was stored at –80°C.

For expression analysis, the cDNA was amplified using following specific primers: *Nrxn1*; sense-TTACTCTGGCTGCTGCAATG, anti-sense-GTCTGAAATCCAGGCCACAT [46], *Nlgn3*; sense-CGTGTATAGCTCTATCCCGGAG, anti-sense- ATTGCTAGCCTCTTCC- TCCTCT [46] and internal control *glyceraldehyde 3-phosphate dehydrogenase* (*GAPDH*); sense-GTCTCCTGCGACTTCAGC, anti-sense-TCATTGTCATACCAGGAAATGA- [47]. The annealing temperature was optimized using gradient RT-PCR amplification from 48 to 64°C and the number of cycles was standardized at optimum temperature from 20–36 cycles. For further experiments, following optimized conditions were used for PCR amplification of *Nrxn1* (94°C for 30 s, 54°C for 30 s, 72°C for 30 s for 28 cycles), *Nlgn3* (94°C for 30 s, 62°C for 45 s, 72°C for 30 s for 28 cycles), and *GAPDH* (94°c for 30 s, 52°C for 30 s, 72°C for 30 s for 26 cycles). The RT-PCR amplicons were run on 2% agarose gel.

### In-situ Hybridization

*In-situ* hybridization was performed as described earlier [48]. Male mice of 3 and 8 weeks were anaesthetized by pentobarbital (50 mg/kgbw, i.p., Sigma Aldrich, USA) as mentioned previously [49] and perfused first with phosphate buffered saline (PBS) and then with 4% paraformaldehyde (PFA). The brain was dissected out and fixed in 4% PFA at 4°C for 12 h. Thereafter, it was immersed in 30% sucrose solution and embedded in optimum cutting temperature (OCT) solution. Transverse 7 µm thick sections were cut by cryostat (MICROM HM 525, Thermo scientific, USA), mounted on poly-L-lysine-coated slides and stored at –80°C for further use. The tissue sections were incubated at 37°C for 15 min, hybridized with digoxigenin (DIG) labeled cDNA probe overnight. The cDNA probes were labeled by PCR using DIG-11-dUTP (Roche, Switzerland), *Nrxn1* and *Nlgn3* specific probes were synthesized using linear pGEM-T-*Nrxn1* and pGEM-T-*Nlgn3* cDNA, respectively. Following hybridization, the tissue sections were washed in 1x sodium saline citrate buffer at 48°C, blocked in 10% goat serum and incubated with horse-radish peroxidase (HRP) conjugated anti-DIG antibody (dilution 1∶2000; Roche, Germany). Detection was done by diaminobenzidine (DAB) method. The slides were examined under a microscope (LEICA DM 2000) and signals were analyzed as mentioned earlier [50].

### Immunoblotting

The cerebral cortex and hippocampus of 3 and 8 weeks male mice were used to prepare 10% homogenate in RIPA buffer [1x PBS, 1% nonyl phenoxypolyethoxylethanol-40, 0.1% sodium dodecyl sulfate (SDS), 0.5% sodium deoxycholate, 100 µg/ml phenylmethanesulfonyl fluoride, 5 µl/100 mg protease inhibitor cocktail].The homogenate was centrifuged at 10,000×g at 4°C for 10 min and supernatant was stored at –80°C until use. The amount of protein in homogenate was estimated [51] and 30 µg protein was denatured, resolved by 10% Tris-glycine SDS-PAGE and transferred onto polyvinylidene fluoride (PVDF) membrane (Millipore, USA). The membrane was blocked in 5% (w/v) nonfat milk prepared in 1x PBS for 3 h at room temperature and incubated overnight with primary antibodies (goat anti Nrxn1, 1∶500; goat anti Nlgn3, 1∶500 and mouse anti β-actin HRP conjugated, 1∶20000) at 4°C. Goat polyclonal Nrxn1 (SC-14093) and Nlgn3 (SC-14334) antibodies were purchased from Santa Cruz Biotechnology (USA), and mouse anti β-actin antibody (A3854) from Sigma Aldrich (USA). After washing thrice (5 min each) in 0.1% PBST (0.1% Tween-20 in 1x PBS), the membrane was incubated with HRP conjugated secondary antibodies obtained from Bangalore Genei, India (rabbit anti goat for both Nrxn1 and Nlgn3, 1∶2000 for 2 h). Finally, the membrane was washed thrice (5 min each) in 0.1% PBST and detected by ECL (Western bright, Advansta, USA) method.

### Immunofluorescence

The brain of 3 and 8 weeks male mice was processed to prepare 7 µm thick transverse sections as described under *in-situ* hybridization method. The sections were fixed in acetone at –20°C for 15 min and rinsed thrice in PBS for 5 min each and incubated with 10% goat serum in 0.1% PBST at room temperature for 2 h to block the non specific sites. Then anti Nrxn1 (1∶50) and anti Nlgn3 (1∶50) primary antibody were added and incubated overnight at 4°C. Primary antibody was not added in negative control slides. Further, the sections were incubated at room temperature for 2 h in tetramethylrhodamine-5/6-isothiocyanate (TRITC) conjugated anti goat IgG (1∶500) for Nrxn1 and fluorescein isothiocyanate (FITC) conjugated anti goat IgG (1∶500) for Nlgn3. Finally, it was rinsed thrice in 1x PBS, mounted in Vectashield mountant containing 4′,6-Diamidino-2-Phenylindole, Dihydrochloride (DAPI) (Vector Laboratories Inc, USA) and detected under a fluorescence microscope using DAPI, TRITC and FITC filters.

### Rapid Golgi Staining

The rapid Golgi staining method was used as described earlier [52]. Male mice of 3 and 8 weeks were deeply anesthetized by pentobarbital (50 mg/kgbw,i.p., Sigma Aldrich, USA) and decapitated quickly. The brain was exposed along midline of the skull and small amount of rapid Golgi fixative (potassium dichromate 5 g, chloral hydrate 5 g, glutaraldehyde 8 ml, formaldehyde 6 ml, dimethylsulfoxide 10 drops/100 ml distilled water) was poured immediately. The brain was dissected out and immersed in amber colored bottle containing 25 ml fixative and kept in dark chamber. On 2^nd^ day, fixative was gently poured out and tissue was rinsed in fresh fixative and again 25 ml fresh fixative was added in the amber bottle. On 3^rd^ day, tissue was again rinsed and 25 ml fresh fixative was added. On 4^th^ day, the tissue was kept undisturbed. Finally, on 5^th^ day, the tissue was rinsed several times in 0.75% AgNO_3_ solution till the reddish brown color of potassium dichromate-silver complex disappeared. Then the tissue was incubated in 25 ml of 0.75% AgNO_3_ solution and kept in dark for 48 h. Finally, 120 µm thick transverse sections were cut by a vibratome (Series-1000), cleared in xylene, mounted on slide using distrene-plasticiser-xylene (DPX) and observed under a microscope.

### Statistical Analysis

All data were analyzed using the software Statistical Package for Social Sciences (SPSS) (version 16). Values were reported as mean ± SEM and *p* values <0.05 were considered as significant. A repeated measures ANOVA was performed for MWM escape latency analysis. Unpaired t-test was performed for probe trial in MWM, RT-PCR, *in-situ* hybridization, immunoblotting, immunofluorescence and rapid Golgi staining. Each molecular experiment was repeated three times (n = 3×3 mice/group). For *Nrxn1* and *NLgn3*, the RT-PCR signal intensity was normalized against *GAPDH* and immunoblotting signal intensity against β-actin. The *in-situ* hybridization and immunofluorescence signal was analyzed by spot densitometry tool of Alpha Ease FC software (Alpha Innotech Corp., USA). Integrated density value (IDV)/unit area of cerebral cortex and dentate gyrus from control and BPA exposed groups were calculated for *Nrxn1* and *Nlgn3* after deducting the value of negative control. The resulting data were analyzed statistically and presented as histograms.

## Results

### Effect of perinatal exposure to BPA on spatial memory of male mice

Morris water maze test was performed to analyze the effect of perinatal BPA exposure on spatial memory of 8 weeks male mice. In this test, control as well as BPA exposed mice showed progressive decline in average escape latency time to find the hidden platform during 8 training days (Fig. 1A). The repeated measures ANOVA showed improvement in performance with training (*F* (7, 140) = 87.641, *p*<0.001). Moreover, a significant interaction was observed between the control and BPA groups during training (*F* (7, 140) = 4.471, *p*<0.001). Further analysis showed statistically significant difference in escape latency between control and BPA groups after day 2 onward. When the path track travelled by mice was traced by ANY-maze software, the BPA exposed group took a longer distance than the control group to find the hidden platform on days of training; the representative data are shown for day 1, 4 and 8 (Fig. 1B). The subsequent probe test after removal of platform on 9^th^ day showed that BPA treated group spent significantly less time in the target quadrant and more time in other quadrants as compared to control group (*p<*0.05) (Fig. 1C, D).Thus the data show clearly that the perinatal exposure to BPA impaired spatial memory of mice.

**Figure 1:** Effect of perinatal exposure to BPA on spatial memory of male mice. Behavior of mice in Morris water maze test to reach the hidden platform. (A) Escape latency (in seconds), (B) Tracking of path on day 1, 4 and 8, (C) Percentage time spent in the target quadrant during probe trial (without platform) and (D) Tracking of path in probe trial. The results are expressed as the mean ± SEM (n = 15 mice/group) and * denotes the significant difference (*p*<0.05) between sesame oil and BPA exposed mice.

### Effect of perinatal exposure to BPA on the expression of Nrxn1 and Nlgn3 in cerebral cortex and hippocampus of male mice

The perinatal exposure to BPA resulted in upregulation of *Nrxn1* and *Nlgn3* mRNA in both cerebral cortex and hippocampus. As compared to control, BPA increased *Nrxn1* mRNA expression significantly in the cerebral cortex (*p*<0.01) and hippocampus (*p*<0.01) of 3 and 8 weeks male mice (Fig. 2A). Similarly, *Nlgn3* mRNA expression was also significantly increased by BPA exposure in the cerebral cortex and hippocampus of 3 and 8 weeks male mice (Fig. 2B). The impact of BPA on the mRNA expression of *Nrx1* and *Nlgn3* was marginally more in hippocampus than cerebral cortex. The effect of BPA exposure persisted even after stopping the treatment, but it was lower in 8 weeks than in 3 weeks. Further, *in-situ* hybridization showed similar pattern of results as observed in RT-PCR in cerebral cortex and dentate gyrus (Fig. 3A, B).

**Figure 2:** Effect of perinatal exposure to BPA on the mRNA expression of Nrxn1 and Nlgn3 in cerebral cortex and hippocampus of male mice. RT-PCR analysis showing mRNA expression of genes following BPA exposure in the cerebral cortex and hippocampus of 3 and 8 weeks male mice (A) *Nrxn1* and (B) *Nlgn3.* Each bar represents the mean ± SEM and * denotes the significant difference (*p*<0.05) between sesame oil and BPA exposed mice.

**Figure 3:** *In-situ* hybridization analysis of Nrxn1 and Nlgn3 mRNA expression upon perinatal exposure to BPA in cerebral cortex and hippocampus of male mice. Photomicrographs of *in-situ* hybridization in cerebral cortex and dentate gyrus of 3 and 8 weeks male mice (A) *Nrxn1* and (B) *Nlgn3*. Histograms represent IDV/Area from three independent experiments. Each bar represents the mean ± SEM and * denotes the significant difference (*p*<0.05) between control and BPA exposed group. Scale bar 50 µm. CC (cerebral cortex) and DG (dentate gyrus).

Nrxn1 was detected as 50 kDa protein, whereas Nlgn3 was detected as 100 kDa protein. Similar to mRNA level, perinatal exposure to BPA resulted in significant upregulation of both Nrxn1 and Nlgn3 protein level (Fig. 4A, B) in cerebral cortex (*p*<0.01) and hippocampus (*p*<0.01) of both 3 and 8 weeks male mice. The effect of BPA also persisted in 8 week mice after abstaining BPA exposure. Immunoblotting result was further supported by immunofluorescence analysis in cerebral cortex and dentate gyrus (Fig. 5A, B).

**Figure 4:** Effect of perinatal exposure to BPA on the expression of Nrxn1 and Nlgn3 proteins in cerebral cortex and hippocampus of male mice. Immunoblotting analysis showing protein expression in the cerebral cortex and hippocampus of 3 and 8 weeks male mice (A) Nrxn1 and (B) Nlgn3. Each bar represents the mean ± SEM and * denotes the significant difference (*p*<0.05) between sesame oil and BPA exposed mice.

**Figure 5:** Immunofluorescence analysis showing BPA induced variation in protein expression of Nrxn1 and Nlgn3 in cerebral cortex and hippocampus of male mice. Photomicrographs of immunofluorescence staining in the cerebral cortex and dentate gyrus of 3 and 8 weeks male mice (A) Nrxn1 (TRITC-labeled) and (B) Nlgn3 (FITC-labeled). Histograms represent IDV/Area from three independent experiments. Each bar represents the mean ± SEM and * denotes the significant difference (*p*<0.05) between sesame oil and BPA exposed mice. Scale bar 100 µm. CC (cerebral cortex) and DG (dentate gyrus).

### Effect of perinatal exposure to BPA on dendritic spine density in cerebral cortex and hippocampus of male mice

The rapid Golgi stain impregnation clearly filled the basilar dendritic shaft and spines of cortical and hippocampal neurons in 3 and 8 weeks male mice. The dendritic spine density was significantly higher in BPA exposed group as compared to control (Fig. 6A, B) in the cerebral cortex (*p*<0.01) and hippocampus (*p*<0.01) of both 3 and 8 weeks male mice. However, the effect of perinatal exposure to BPA was higher in hippocampus as compared to cerebral cortex. The increased number of dendritic spines persisted even after the BPA exposure was stopped.

**Figure 6:** Effect of perinatal exposure to BPA on dendritic spine density in cerebral cortex and hippocampus of male mice. Rapid Golgi staining of neurons in the cerebral cortex and hippocampus of 3 and 8 weeks male mice. The histograms represent the number of dendritic spines/10 µm length of primary dendrites. Each bar represents the mean ± SEM of 15 neurons from three independent experiments and * denotes the significant difference (*p*<0.05) between sesame oil and BPA exposed mice.

## Discussion

It has been well established that certain periods during development such as embryonic stage, early postnatal life and juvenile stage are critically susceptible to BPA exposure [53]. The levels of endogenous hormones all through the developmental period are essential for regulating the sexual differentiation of brain and behavior [54]. Growing body of studies has established the effect of perinatal exposure to BPA on memory impairment [13], [55]. However, the effect of perinatal exposure on synaptic plasticity proteins, which play a key role in memory, is poorly understood.

The present study showed that the escape path length in water maze extended while the percentage of time spent in the target quadrant decreased by perinatal exposure to BPA in 8 weeks male mice. An earlier study also reported that the perinatal BPA exposure within the range of human exposure impaired the spatial memory of male offspring in MWM test [41]. Other studies also showed that BPA impaired various behavioral paradigms in rodents such as exploratory behavior [13], sociosexual behavior [14] and memory [18]. Taken together, these data showed that perinatal exposure to BPA impaired spatial memory in male mice.

The basis of learning and memory is formation of synapse which begins in the embryo and continues to early postnatal life and adults [56]. Synapse formation involves several steps including neurite outgrowth, contact initiation, recruitment of pre and postsynaptic proteins and their stabilization [57]. Several studies have suggested that synaptic proteins Nlgns and Nrxns play an important role during the initial step of synaptogenesis [28], [29], [58]. Moreover, in non-neuronal cells, Nlgns triggered presynaptic development in adjoining axons [59]. Similarly, Nrxns induced differentiation of GABAergic and glutamatergic postsynaptic specialization in non-neuronal cells [34]. Deletion of Nrxns causes a major decrease in action potential evoked by neurotransmitter release and a massive impairment in Ca^2+^ channel function [60]. In addition, Nrxns and Nlgns are linked to synaptic functions in cognitive diseases [38]. Their interaction is involved in neuronal plasticity mechanisms and neuronal disorders such as autism [38]. In humans, more than 30 *Nlgns* gene mutations have been associated with autism, including *Nlgn3* point mutation [61] and deletion [62]. We have observed upregulation of Nrxn1 and Nlgn3 mRNA and protein expression in both cerebral cortex and hippocampus of BPA exposed 3 and 8 weeks male mice as compared to control. As the over-expression of Nlgn1 or Nlgn2 in neuronal culture increased the number of excitatory and inhibitory synapses [63], it is likely that BPA mediated upregulation of Nrxn1 and Nlgn3 might be involved in altering the ratio of excitatory/inhibitory synapse. A mismatch of Nrxns and Nlgns partner in honey bee across synapse in the brain presumably leads to loss of synaptic plasticity and/or erroneous wiring of synapses, resulting in behavioral and cognitive deficiencies [64].

Almost all the fast synaptic activity in the cortex is mediated by the glutamatergic excitatory and GABAergic inhibitory synapses [65]. The excitatory inputs and local excitatory transmission in the cortex play a crucial role in the acquisition, consolidation and retrieval of spatial memory [66]. The principal neurons in the superficial layers of medial entorhinal cortex receive visuospatial information from the neocortex primarily through excitatory synapses and then transfer the information to all the sub-regions of hippocampus [67], [68]. Studies suggest that dendritic spines are the primary recipient of excitatory inputs and play an important role in determining neuronal input-output transformation [69]. Our findings showed that perinatal exposure to BPA increased dendritic spine density in cerebral cortex and hippocampus of 3 and 8 weeks male mice. Such changes in spine number might disrupt the neural circuitry and alter the firing properties of functional neurons, leading to impairment of memory. As reported earlier, acute exposure to BPA in ovariectomized mice blocked the estrogen induced memory enhancement [70]. Moreover, perinatal exposure to BPA inhibited synaptogenesis and affected the synaptic development in male mice [21].

In conclusion, the present study shows that the upregulation of expression of synaptic proteins Nrxn1 and Nlgn3 might be involved in BPA mediated dysregulation of learning and memory, which could be mediated through the increase in dendritic spine density that might disrupt the delicate balance between excitatory and inhibitory synapse, or form erroneous wiring of synapses in the brain.
